This article has been retracted.

# ErbB4 Preserves Blood-Brain Barrier Integrity via the YAP/PIK3CB Pathway After Subarachnoid Hemorrhage in Rats

**DOI:** 10.3389/fnins.2018.00492

**Published:** 2018-07-24

**Authors:** Huan Qian, Zhangqi Dou, Wu Ruan, Pingyou He, John H. Zhang, Feng Yan

**Affiliations:** ^1^Department of Plastic Surgery, The Second Affiliated Hospital, School of Medicine, Zhejiang University, Hangzhou, China; ^2^Department of Neurosurgery, The Second Affiliated Hospital, School of Medicine, Zhejiang University, Hangzhou, China; ^3^Division of Physiology, Department of Basic Sciences, Loma Linda University School of Medicine, Loma Linda, CA, United States

**Keywords:** ErbB4, YAP, PIK3CB, blood-brain barrier, early brain injury, subarachnoid hemorrhage

## Abstract

Studies have suggested that blood-brain barrier (BBB) disruption contributes to the pathogenesis of early brain injury after subarachnoid haemorrhage (SAH). Activation of the receptor tyrosine kinase ErbB4 can cause intramembrane proteolysis and release a soluble intracellular domain (ICD) that modulates transcription in the nucleus. This study was carried out to investigate the potential roles of ErbB4 in preserving BBB integrity after experimental SAH, as well as the underlying mechanisms of its protective effects. Endovascular perforation was used to prepare a rat SAH model. The SAH grade, neurological score, brain edema and BBB permeability were evaluated after surgery. Immunohistochemistry was used to determine the localization of ErbB4 and yes-associated protein (YAP). ErbB4 activator Nrg1 isoform β1 (Nrg1β1), Specific ErbB4 siRNA, YAP siRNA and PIK3CB specific inhibitor TGX 221 were used to manipulate the proposed pathway. The expression levels of ErbB4 ICD and YAP were markly increased after SAH. Double immunohistochemistry labeling showed that ErbB4 and YAP were expressed in endothelial cells and neurons. Activation of ErbB4 by Nrg1β1 (dosage 150 ng/kg) treatment promoted the neurobehavioral deficit, alleviated the brain water content and reduced albumin leakage 24 and 72 h after SAH. ErbB4 activation significantly promoted YAP and PIK3CB activity and increased the expression of tight junction proteins Occludin and Claudin-5. Depletion of ErbB4 aggravated neurological impairment and BBB disruption after SAH. The beneficial effects of ErbB4 activation were abolished by YAP small-interfering RNA and specific PIK3CB inhibitor. Activation of ErbB4 improved neurological performance after SAH through the YAP/PIK3CB signaling pathway, this neuroprotective effects may associated with BBB maintenance.

## Introduction

Aneurysmal subarachnoid hemorrhage (SAH) is one of the most life-threatening diseases, with high mortality and disability rates (Connolly et al., 2012). Recent studies have shifted the research focus from SAH-induced vasospasm to early brain injury. Defined as the pathophysiological event that occurs within 72 h after SAH, early brain injury (EBI) has been proposed as the primary determinant of poor outcome in SAH patients (Sehba et al., 2012). Nevertheless, the definitive mechanisms of EBI after SAH have remained unclear, and blood-brain barrier (BBB) disruption plays an important role (Chen et al., 2014; Li et al., 2015). Strategies against BBB disruption after SAH may be helpful in attenuating EBI and lead to a better prognosis.

ErbB4 (EGFR family member v-erb-b2 avian erythroblastic leukemia viral oncogene homolog 4) is a kind of epidermal growth factor receptor kinases, which has been proven to play a key role in the regulation of neurite outgrowth, axonal guidance and synaptic signaling (Huang et al., 2000; Shamir et al., 2012). ErbB4 can undergo intramembrane proteolysis to release a soluble intracellular domain (ICD) (Ni et al., 2001). The ErbB4 ICD relocalizes to the nucleus, where it regulates transcription through its association with transcriptional co-regulators (Vidal et al., 2005; Gilmore-Hebert et al., 2010). Mice lacking ErbB4 receptor have shown defects in axon guidance in the central nervous system (Tidcombe et al., 2003). In an oxidative stress injury study, ErbB4 promoted the survival of endothelial cells and preserved BBB integrity (Lok et al., 2009). However, the precise role of ErbB4 during the pathological process after subarachnoid hemorrhage (SAH) and its acting pathway remain largely unknown.

ErbB4 was found to be a major receptor that could activate Yes-associated protein (YAP), which has emerged as a critical signaling hub that regulates cellular growth and organ size maintenance (Dong et al., 2007). Activation of YAP stimulated the expression of genes that contribute to cellular development (Zhao et al., 2010). PIK3CB is a catalytic component of phosphoinositol-3-kinase (PI3K), which was reported to be activated downstream of YAP (Lin et al., 2015). This study investigated potential effects of ErbB4 with its downstreams on BBB integrity in EBI after SAH.

## Materials and Methods

### Study Design

All procedures were conducted following the institutional Animal Care and Use Committee at Zhejiang University and in accordance with NIH guidelines for the Care and Use of Laboratory Animals. Two hundred and eight three Male Sprague-Dawley (SD) rats (290–330 g; Harlan, Indianapolis, IN, United States) were housed in a humidity-controlled room (25 ± 1°C, 12-h light/dark cycle) and were raised with free access to water and food.

#### Experiment 1

To detect the time course expressions of ErbB4 and YAP in the sham group and at 3, 6, 12, 24, and 72 h after SAH (*n* = 6 in each group). Double immunohistochemistry staining of ErbB4/YAP with CD31 was performed at 24 h after SAH (*n* = 2) for morphological study.

#### Experiment 2

Extracellular domain of Neuregulin 1 isoformβ1 (Nrg1β1, R&D systems, Minneapolis, MN, United States) was used for activation of ErbB4, and administered intraperitoneally at 1 h after SAH induction. Besides the sham and vehicle groups, two groups of rats received a different dosage of Nrg1β1 (50 ng/kg and 150 ng/kg, *n* = 6). The dose of Nrg1β1was set according to a previous study (Depboylu et al., 2015). For outcome evaluation, neurobehavioral scores, brain edema and albumin extravasation were measured at 24 and 72 h after SAH in all groups (*n* = 6). The expression levels of ErbB4, ErbB4 ICD, YAP, PIK3CB, Occludin and Claudin-5 were analyzed via Western blotting.

#### Experiment 3

ErbB4 small-interfering RNA (siRNA) was injected via intracerebroventricular (ICV) administration at 24 h before SAH induction. The neurobehavior, brain edema, albumin extravasation and expression of ErbB4, YAP, PIK3CB, Occludin and Claudin-5 were measured at 24 h after SAH in all groups. The rats were randomly assigned into the following groups: SAH + Vehicle, SAH + Nrg1β1, SAH + Nrg1β1 + scrambled siRNA (in 5 μl sterile saline), and SAH + Nrg1β1 + ErbB4 siRNA (in 5 μl of sterile saline).

#### Experiment 4

Yes-associated protein siRNA was administered by ICV injection at 24 h before SAH. Neurobehavior, brain edema, albumin extravasation and the expression levels of ErbB4, YAP, PIK3CB, Occludin, and Claudin-5 were measured at 24 h after SAH in all groups. Rats were randomly assigned into the following groups: SAH + Vehicle, SAH + Nrg1β1, SAH + Nrg1β1 + scrambled siRNA (in 5 μl of sterile saline), and SAH + Nrg1β1 + YAP siRNA (in 5 μl of sterile saline).

#### Experiment 5

The PIK3CB specific inhibitor TGX 221 (2.5 mg/kg, I.V., Cayman Chemical Corp., Ann Arbor, MI, United States) dissolved in PBS was administered at 1 h before SAH induction (Sturgeon et al., 2008). Control animals were injected with the same volume of PBS. Neurobehavior, brain edema, BBB permeability and western blots were measured at 24 h after SAH in all groups.

### SAH Model

The SAH rat model was induced by endovascular perforation as previously described (Yan et al., 2017a). The rats underwent tracheal intubation with 3% isoflurane anesthesia. Next, we dissected the left external carotid artery, and a sharpened, 4-0 monofilament nylon suture was inserted vertically into the left internal carotid artery through the bifurcation of the external carotid artery until we felt slight resistance. The suture was then further advanced to impale the vessel. Sham-operated rats underwent nearly the same procedure, and we withdrew the suture once resistance was felt without any puncture.

### Intracerebroventricular Drug Injection

Intracerebroventricular drug injection was performed as reported previously (Yan et al., 2017b). The rats were placed in a stereotaxic apparatus under 2.5% isoflurane anesthesia. The needle of a 10-μl Hamilton syringe (Microliter701; Hamilton Company, Reno, NV, United States) was stereotactically inserted through a burr hole into the left lateral ventricle, which is coordinated relative to the bregma as follows: 1.5 mm posterior, 1.0 mm lateral and 3.5 mm below the horizontal plane of the skull. Next, 500 pmol/5 μl of ErbB4 siRNA (Thermo Fisher Scientific, Waltham, MA, United States), YAP siRNA (Thermo Fisher Scientific, Waltham, MA, United States), or scrambled siRNA (Thermo Fisher Scientific, Waltham, MA, United States) was injected at 1 day before SAH induction with Lipofectamine 2000 (Thermo Fisher Scientific, Waltham, MA, United States) at the rate of 0.5 μl/min. To enhance the gene silencing efficiency, two different ErbB4 siRNAs were mixed (5′ CCCACUAGUCAUGACUGCAUUUACU3′ and 5′AGUAAAUGCAGU-CAUGACUAGUGGG3′) and two different YAP siRNAs were mixed (5′GGCUGC-GAUUGAAACAGCAGGAGUU3′ and 5′AACUCCUGCUGUUUCAAUCGCAGC-C3′).

### SAH Grade

The severity of SAH was quantified using a previously published grading scale at the time of euthanasia (Sugawara et al., 2008). The basal cistern was divided into 6 segments, and the amount of the subarachnoid blood clot on each segment was scored from 0 to 3. Each rat received a total SAH score ranging from 0 to 18, and rats with mild SAH (score < 8) were excluded from this study.

### Neurological Score

Neurological deficits were evaluated at 24 and 72 h after SAH according to the modified Garcia’s scoring system (Garcia et al., 1995): spontaneous activity, symmetry in movement of four limbs, forepaw outstretching, climbing, body proprioception, and response to vibrissae touch. The total scores of the modified Garcia’s test ranged from 3 to 18. Additionally, beam balance test (4-point scoring system) was performed (Tang et al., 2015). The rats were placed on a beam, and the walking distance within 1 min was measured (0–4).

### Brain Water Content

The brains were collected 24 and 72 h after SAH induction and were separated into the left hemisphere, right hemisphere, cerebellum and brain stem. Each part was weighed immediately after removal (wet weight) and then was dried in an oven at 105°C for 72 h before another weighing (dry weight). The percentage of water content was calculated following the equation: [(wet weight- dry weight)/wet weight] × 100% (Chen et al., 2015).

### Immunofluorescence Staining

Double-immunofluorescence staining of cerebral cortex was performed at 24 h after SAH as described previously (Xie et al., 2017). Sections were incubated overnight at 4°C with rabbit anti-ErbB4 (Abcam, Cambridge, MA, United States), rabbit anti-YAP (Cell Signaling Technology, Beverly, MA, United States), and mouse anti-CD31 (Abcam, Cambridge, MA, United States), followed by fluorescence dye-conjugated secondary antibodies (Jackson Immunoresearch, West Grove, PA, United States) for 3 h at 20°C. The sections were then visualized with a fluorescence microscope. Photomicrographs were analyzed using Image-Pro Plus software (Olympus, Melville, NY, United States).

### Western Blotting

Western blot analysis was performed as previously described (Yan et al., 2014). The left brain hemisphere (perforation side) was collected according to scheduled time point. Equivalent amounts of protein (50 μg) were loaded onto sodium dodecyl sulfate (SDS) polyacrylamide gels and were separated by electrophoresis. The proteins were transferred onto nitrocellulose membranes, which were blocked by a blocking buffer. Primary antibodies were diluted to incubate with the membrane under gentle agitation at 4°C overnight: anti-ErbB4 (Abcam, Cambridge, MA, United States), anti-YAP (Cell Signaling Technology, Beverly, MA, United States), anti-PIK3CB (Abcam, Cambridge, MA, United States), anti-Occludin (Abcam, Cambridge, MA, United States), anti-Claudin-5 (Thermo Fisher Scientific, Waltham, MA, United States) and anti-β-actin (Santa Cruz Biotechnology, Dallas, TX, United States). Appropriate secondary antibodies were incubated with the membrane for 2 h at room temperature. Chemiluminescent detection was performed to identify the immune bands using the ECL Plus kit (Amersham Bioscience, Arlington Heights, IL, United States). Data was analyzed by densitometry with Image J software.

### Statistical Analysis

One-way ANOVA followed by Turkey’s multiple comparisons test was used for comparison between groups. The data were expressed as means ± SEM. *P* < 0.05 was considered statistically significant. All statistical analyses were performed using GraphPad Prism for Windows (LaJolla, CA, United States).

## Results

### Mortality and Exclusion

There was no significant difference in the SAH grading score in all SAH groups (**Supplementary Figures S1A,B**). No rats died in the sham group. The mortality rate for each group is listed as follows: SAH group 18.18% (8/44), SAH + Vehicle group 21.43% (9/42), SAH + Nrg1β1 (50 ng/kg) group 17.07% (7/41), SAH + Nrg1β1 (150 ng/kg) group 13.51% (5/37), SAH + Nrg1β1 + Scr siRNA group 13.33% (2/15), SAH + Nrg1β1 + ErbB4 siRNA group 22.22% (4/18), SAH + Nrg1β1 + Scr siRNA group 14.29% (2/14), SAH + Nrg1β1 + YAP siRNA group 23.53% (4/17), SAH + Nrg1β1 + TGX 221 group 26.32% (5/19) (**Supplementary Figure S1C**). According to the SAH grading score, 19 rats with mild SAH were excluded from this study (**Supplementary Table S1**).

### Time Course of Endogenous ErbB4, ErbB4 ICD and YAP Expression After SAH

Western blot analysis was applied on the rats of all groups at different time points after SAH induction (**Figure 1A**). The results demonstrated a significant increasing in the expression of ErbB4 ICD as early as 3 h after SAH. This trend continued and reached a peak at 72 h after SAH, while the total ErbB4 level remained stable (*p* < 0.05, **Figure 1B**). A similar tendency was observed in the expression of YAP, which started to increase at 3 h after SAH (*p* < 0.05, **Figure 1C**). Morphological study with double immunohistochemistry staining showed that ErbB4 expression was colocalized with CD31 (Marker for endothelial cell), YAP was also proved to be intensely expressed in CD31-positive cells (**Figure 1D**). Double immunostaining showed that both ErbB4 and YAP were colocalized with Neuron at 24 h after SAH (**Supplementary Figure S2**).

**FIGURE 1:** Expression of endogenous ErbB4, ErbB4 ICD and YAP after subarachnoid haemorrhage (SAH) induction. Representative Western blot bands of ErbB4, ErbB4 ICD and YAP from the ipsilateral hemisphere after SAH **(A)**, quantitative analyses of ErbB4 ICD/ErbB4 **(B)** and YAP **(C)** expression. *n* = 6. Double immunostaining showed that both ErbB4 and YAP were colocalized with CD31-positive endothelial cells at 24 h after SAH **(D)**. *n* = 2, ^∗^*p* < 0.05 versus sham; #*p* < 0.05 versus 72 h.

### Nrg1β1 Treatment Improves Neurobehavioral Functions and Reduces BBB Permeability After SAH

Remarkable neurobehavioral impairment was observed in the vehicle and Nrg1β1 (50 ng/kg)-treated group compared with that in the sham group at 24 and 72 h after SAH. Post-SAH administration of high-dosage Nrg1β1 (150 ng/kg) significantly improved the neurobehavioral performance (*p* < 0.05, **Figures 2A,B**). Brain water content in both hemispheres significantly increased in rats from the vehicle and Nrg1β1 (50 ng/kg)-treated group at 24 and 72 h after SAH (*p* < 0.05, **Figures 2C,E**). Nrg1β1 (150 ng/kg) treatment significantly decreased brain water content and attenuated brain swelling compared with the vehicle and Nrg1β1 (50 ng/kg) -treated group (*p* < 0.05, **Figures 2C,E**). BBB permeability was assessed by albumin extravasation in the ipsilateral hemisphere. Western blot analysis demonstrated a remarkable increased expression of albumin in vehicle and Nrg1β1 (50 ng/kg)-treated rats at 24 and 72 h after SAH that was significantly reversed by Nrg1β1 (150 ng/kg) treatment (*p* < 0.05, **Figures 2D,F**).

**FIGURE 2:** Neuregulin1 isoformβ1 (Nrg1β1) treatment improved neurological functions, reduced brain water content and deceased albumin leakage at 24 and 72 h after SAH. Neurological impairment **(A,B)**, increased brain water content **(C,E)** and albumin extravasation **(D,F)** were found in the SAH + Vehicle groups. Nrg1β1 (150 ng/kg) treatment significantly alleviated neurological deficit **(A,B)**, reduced brain water content **(C,E)** and deceased albumin extravasation **(D,F)**. *n* = 6 for each group. ^∗^*p* < 0.05 versus sham; #*p* < 0.05 versus SAH + vehicle; &*p* < 0.05 versus SAH + Nrg1β1 (50 ng/kg).

### ErbB4 Activation by Nrg1β1 Administration Stabilizes Tight Junction Proteins After SAH

The expression of ErbB4 and its downstream signals was measured by western blot analysis (**Figure 3A**). The ratio of ErbB4 ICD/ErbB4 expression significantly increased after Nrg1β1 (50 ng/kg) administration and was further increased by high-dose Nrg1β1 (150 ng/kg) treatment compared with that in the sham and vehicle group (*p* < 0.05, **Figure 3B**). The expression level of YAP and PIK3CB was also significantly upregulated after Nrg1β1 administration, and there was a significant dose-dependent effect (*p* < 0.05, **Figures 3C,D**). The expression levels of tight junction proteins Occludin and Claudin-5 were significantly reduced at 24 h after SAH in the vehicle and low-dose Nrg1β1 (50 ng/kg)-treatment group. Treatment of Nrg1β1 (150 ng/kg) significantly reversed this tendency (*p* < 0.05, **Figures 3E,F**).

**FIGURE 3:** ErbB4 activation by Nrg1β1 administration stabilizes tight junction proteins. Representative western blot bands of ErbB4, YAP, PIK3CB, Occludin and Claudin 5 **(A)**, the expression of ErbB4 ICD/ErbB4 **(B)**, YAP **(C)**, and PIK3CB **(D)** were increased at 24 h after SAH induction and were further up-regulated by high-dose Nrg1β1 (150 ng/kg) administration. SAH induction significantly reduced the expression of Occludin **(E)** and Claudin-5 **(F)**. Nrg1β1 (150 ng/kg) administration significantly reversed this effect. *n* = 6, ^∗^*p* < 0.05 versus sham; #*p* < 0.05 versus SAH + vehicle; &*p* < 0.05 versus SAH + Nrg1β1 (50 ng/kg).

### Silencing ErbB4 Aggravates Neurological Deficits and BBB Disruption After SAH

ErbB4 knockdown by siRNA significantly aggravated neurological deficits and increased albumin extravasation at 24 h after SAH (*p* < 0.05, **Figures 4A,B**) compared with that in the Nrg1β1-treatment group. The silencing efficacy of ErbB4 with its downstream signals and their effects on tight junction protein expression was measured by western blotting analysis (**Figure 4C**). Injection of scrambled siRNA had no effect on the expression of ErbB4 after Nrg1β1 administration (*p* > 0.05, **Figure 4D**), while specific ErbB4 siRNA significantly decreased the ratio of ErbB4 ICD/ErbB4 (*p* < 0.05, **Figure 4D**). ErbB4 activation promoted YAP expression with its downstream protein PIK3CB, which were both remarkably decreased by ErbB4 siRNA administration (*p* < 0.05, **Figures 4E,F**). The increased expression of Occludin and Claudin-5 after Nrg1β1 treatment was significantly reversed by ErbB4 siRNA injection (*p* < 0.05, **Figures 4G,H**).

**FIGURE 4:** Effects of ErbB4 siRNA pre-treatment on blood-brain barrier integrity at 24 h after SAH. ErbB4 siRNA aggravated neurological deficits **(A)** and increased albumin extravasation **(B)**. Representative western blot bands of ErbB4, YAP, PIK3CB, Occludin and Claudin 5 **(C)**. ErbB4 knockdown decreased the expression of ErbB4 ICD/ErbB4 **(D)**, YAP **(E)**, and PIK3CB **(F)**. The increased expression levels of Occludin and Claudin-5 after Nrg1β1 treatment were significantly reduced by ErbB4 depletion **(G,H)**. The PIK3CB specific inhibitor TGX 221 did not affect the expression of ErbB4 ICD/ErbB4 **(D)**, YAP **(E)** and significantly reduced the expression of PIK3CB **(F)**, Occludin **(G)** and Claudin-5 **(H)**. *n* = 6, #*p* < 0.05 versus SAH + vehicle; @*p* < 0.05 versus SAH + Nrg1β1; §*p* < 0.05 versus SAH + Nrg1β1 + ErbB4siRNA.

### YAP Knockdown Reversed the Protective Effects of ErbB4 Activation on BBB Integrity After SAH

Subarachnoid haemorrhage rats were administered scrambled or YAP-specific siRNA before Nrg1β1 treatment to further explore the downstream signaling pathway participating in ErbB4 activation. YAP depletion significantly aggravated neurological deficits and increased albumin extravasation at 24 h after SAH (*p* < 0.05, **Figures 5A,B**). Western blot analysis was used to measure the effects of YAP knockdown and PIK3CB inhibition on tight junction protein expression (**Figure 5C**). Both scrambled and YAP siRNA injection had no effect on the increased ratio of ErbB4 ICD/ErbB4 expression after Nrg1β1 administration (*p* > 0.05, **Figure 5D**). YAP knockdown by specific siRNA significantly reduced the expression of YAP and its downstream PIK3CB (*p* < 0.05, **Figures 5E,F**). The expression level of tight junction protein Occludin and Claudin-5 were highly preserved by Nrg1β1 treatment at 24 h after SAH, but this tendency was significantly abolished by YAP siRNA pre-administration (*p* < 0.05, **Figures 5G,H**).

**FIGURE 5:** Effects of YAP siRNA pre-treatment on blood-brain barrier integrity at 24 h after SAH. YAP siRNA aggravated neurological deficits **(A)** and increased albumin extravasation **(B)**. Representative western blot bands of ErbB4, YAP, PIK3CB, Occludin and Claudin 5 **(C)**. YAP knockdown did not affect the ratio of ErbB4 ICD/ErbB4 **(D)**, and reduced the expression of YAP **(E)**, PIK3CB **(F)**, Occludin **(G)**, and Claudin-5 **(H)**. PIK3CB inhibition by TGX 221 had no effect on the expression of ErbB4 ICD/ErbB4 **(D)** and YAP **(E)**, and significantly reduced the expression of PIK3CB **(F)**, Occludin **(G)** and Claudin-5 **(H)**. *n* = 6, #*p* < 0.05 versus SAH + Vehicle; @*p* < 0.05 versus SAH + Nrg1β1; *p* < 0.05 versus SAH + Nrg1β1 + YAP siRNA.

### Inhibition of PIK3CB Reverses the Beneficial Effects of erbB4 Activation on BBB Integrity After SAH

The potent PIK3CB inhibitor TGX 221 significantly aggravated neurological deficits and increased albumin extravasation at 24 h after SAH (*p* < 0.05, **Figures 4A,B**). Western blotting indicated that TGX 221 injection did not affect the ratio of ErbB4 ICD/ErbB4 and YAP expression (*p* > 0.05, **Figures 4D,E**) but remarkly reduced PIK3CB expression (*p* < 0.05, **Figures 4F**, **5F**). The increased expression of tight junction protein Occludin and Claudin-5 by Nrg1β1 treatment was significantly reversed by TGX 221 administration (*p* < 0.05, **Figures 4G,H**, **5G,H**).

## Discussion

In the present study, we elucidated the ErbB4-mediated signaling pathway in BBB protection following SAH in rats. This study demonstrated a significant increase in the expression of ErbB4 ICD and YAP in the rat brain within 72 h after SAH. Double-immunofluorescence staining indicated that both ErbB4 and YAP were expressed in endothelial cells. Activation of ErbB4 by recombinant Nrg1β1 treatment improved the neurological deficit, reduced brain edema and alleviated BBB disruption after SAH, which were associated with increased expression of tight junction protein Occludin and Claudin 5. Specific siRNA injection eliminated the protective effects of ErbB4 activation after SAH induction, accompanied by the reduction of YAP and PIK3CB expression. YAP siRNA administration reversed the protective effects of ErbB4 activation with reduced downstream signal expression. The neuroprotective effects of ErbB4/YAP/PIK3CB signaling activation was significantly abolished by PIK3CB inhibition, with degraded tight junction proteins and increased BBB disruption. These data indicated that ErbB4 has great effects on maintaining BBB integrity and ameliorating EBI after SAH in rats, possibly through the YAP/PIK3CB signaling pathway.

ErbB4 is one of the epidermal growth factor receptor tyrosine kinase (RTKs) family, which has great effects on neural development and differentiation. ErbB4 is unusual among RTKs in its ability to undergo regulated intramembrane proteolysis to release a soluble ICD (Ni et al., 2001). The ErbB4 ICD relocalizes to the nucleus, where it regulates transcription through its association with transcriptional co-regulators (Vidal et al., 2005; Gilmore-Hebert et al., 2010). Recent studies have suggested that ErbB4 plays an essential role in the regulation of neurite outgrowth, axonal guidance and synaptic signaling (Huang et al., 2000; Shamir et al., 2012). Previous studies have proven that mice lacking ErbB4 receptor could show defects in axon guidance in the central nerves system (Tidcombe et al., 2003). Upregulated ErbB4 expression helps to protect against neuronal cell apoptosis after brain ischaemia (Lu et al., 2016). ErbB4 was found to promote the survival of endothelial cells and preserve BBB integrity (Lok et al., 2009) in a study about oxidative stress injury. In this study, we found that ErbB4 activation significantly alleviated neurological deficits, reduced brain edema and alleviated BBB disruption after SAH. Increased expression of tight junction proteins Occludin and Claudin-5 were observed after ErbB4 activation, which was accompanied by improved BBB integrity after SAH. ErbB4 blockage by specific siRNA could significantly reverse these beneficial effects and aggravate BBB disruption. These findings suggested the protective effects of ErbB4 on maintaining BBB integrity after SAH.

The transcriptional co-activator YAP was found to be essential for cell proliferation as a nuclear effecter of the Hippo-kinase cascade, which is a critical signaling hub that regulates organ growth and size maintenance. Studies have showed that YAP regulates the expression of target genes manipulate DNA transcription (Zhao et al., 2010). Once activated, YAP stimulated fetal and adult cardiomyocyte proliferation (Lin et al., 2015). In the past decade, many components of the Hippo pathway were discovered by Drosophila mosaic genetic screens and proved to be highly conserved in mammals (Low et al., 2014). Among them, YAP was confirmed to be functional in organ size regulation and tumourigenesis in mammals as a directly phosphorylated transcription co-activator. A study by Haskins et al. provided compelling evidence that ErbB4 and its activator Nrg1β1 robustly regulate the Hippo-YAP pathway. Elevation of ErbB4 in cultured mammary epithelial cells promoted the expression of genes regulated by YAP, implying ErbB4-YAP signaling might exist in mammals (Haskins et al., 2014). In this study, activation of ErbB4 significantly increased YAP expression. Knockdown of ErbB4 by specific siRNA significantly down-regulated the expression level of YAP and its downstream signals. Meanwhile, YAP blockage by specific siRNA abolished protective effects of ErbB4 activation, aggravated neurological deficits and BBB disruption, and degraded tight junction expression without affecting ErbB4 expression. These results suggested that the protective role of ErbB4 in maintaining BBB integrity after SAH may be mediated by YAP.

PIK3CB is an p110 catalytic component of Class IA PI3Kwhich has been found to be directly regulated by YAP (Ilic and Roberts, 2010; Lin et al., 2015). YAP has been reported to increase the expression of PIK3CB, and promote cardiomyocyte survival (Lin et al., 2015). The present study demonstrated that the activation of ErbB4 significantly enhanced the expression of YAP and PIK3CB and improved BBB integrity after SAH. Knockdown of ErbB4 or YAP by specific siRNA significantly reduced PIK3CB expression and aggravated BBB disruption. PIK3CB inhibition by TGX 221 significantly reversed the beneficial effects of ErbB4 activation, aggravated neurological deficits and BBB disruption, and degraded tight junction expression without affecting the expression of ErbB4 and YAP.

There are some limitations in this study. Double-immunofluorescence staining indicated that ErbB4 and YAP both expressed in neuron and endothelial cells, which implied that ErbB4 signaling activation could protect against SAH in multiple ways besides BBB maintenance. Previous study have demonstrated the anti-apoptotic effects of ErbB4 in endothelial cells (Lok et al., 2009). Our study showed strong expression of ErbB4 and YAP in neurons, which implied that ErbB4 activation may effects neuron survival after SAH. This hypnosis needs further exploration. In conclusion, this study demonstrated that activation of ErbB4 could improve neurological impairment and reduce brain edema after SAH via the YAP/PIK3CB signaling pathway, this effects may associated with and preserved BBB integrity.

## Author Contributions

HQ and FY conceived and designed the study, including quality assurance and control. ZD and WR performed the experiments and wrote the paper. PH designed the study’s analytic strategy. JZ helped conduct the literature review. All the authors read and approved the manuscript.

## Conflict of Interest Statement

The authors declare that the research was conducted in the absence of any commercial or financial relationships that could be construed as a potential conflict of interest.

## Supplementary Material

FIGURE S1 Representative Photograph of SAH model, SAH grading and mortality among each group. **(A)** Representative photographs of sham and SAH model. **(B)** There was no significant difference of SAH grading among all the experimental groups. **(C)** The mortality for each group are listed as follow: The mortality rate for each group is listed as follows: SAH group 18.18% (8/44), SAH + Vehicle group 21.43% (9/42), SAH + Nrg1β1 (50 ng/kg) group 17.07% (7/41), SAH + Nrg1β1 (150 ng/kg) group 13.51% (5/37), SAH + Nrg1β1 + Scr siRNA group 13.33% (2/15), SAH + Nrg1β1 + ErbB4 siRNA group 22.22% (4/18), SAH + Nrg1β1 + Scr siRNA group 14.29% (2/14), SAH + Nrg1β1 + YAP siRNA group 23.53% (4/17), SAH + Nrg1β1 + TGX 221 group 26.32% (5/19). No statistically significant difference was observed among all the operated groups.

FIGURE S2 Immunofluorescence double staining of ErbB4 (red), YAP (red), and neuronal marker (NeuN, green) showed that the expression of ErbB4 and YAP were localized in neurons at 24 h after SAH. *n* = 2, bars = 100 μm.

TABLE S1 Numbers of animals used in each group.
